This article has been retracted.

# The Neuroprotective Effect of miR-136 on Pilocarpine-Induced Temporal Lobe Epilepsy Rats by Inhibiting Wnt/*β*-Catenin Signaling Pathway

**DOI:** 10.1155/2022/1938205

**Published:** 2022-02-26

**Authors:** Hongxia Cui, Weihao Zhang

**Affiliations:** Department of Neurology, Changzhou Hospital District, 904 Hospital of PLA Joint Logistics Support Force, Changzhou, Jiangsu 213003, China

## Abstract

**Objective:**

To explore the effect of miR-136 on temporal lobe epilepsy (Ep) and its mechanism of action.

**Methods:**

30 male rats were injected intraperitoneally with 30 mg/kg pilocarpine to construct a rat temporal lobe epilepsy model, and they were randomly divided into 5 groups (*n* = 6 per group): control group, Ep group, agomir NC group, miR-136 agomir group, and miR-136+LiCl group. The brain tissues of the rats were collected 7 days after the treatment. The expression of miR-136 in the hippocampus tissue was detected by qRT-PCR. H&E and Nissl staining were used to observe the histopathological changes and neuron damage in the hippocampus tissue. IL-1*β*, IL-6, and TNF-*α* levels in the hippocampus tissue were detected by ELISA. Flow cytometry was used to detect the apoptosis rate in the hippocampus tissue. Western blot was used to detect the expression levels of c-Caspase-3, Bcl-2, *β*-catenin, Cyclin D1, and c-myc protein in the hippocampus.

**Results:**

The expression of miR-136 was significantly downregulated in the hippocampus tissue of epileptic rats. After overexpression of miR-136, the number of seizures and the duration of epilepsy in rats were significantly reduced. At the same time, hippocampal tissue damage was improved considerably, and the degree of neuronal damage decreased. Overexpression of miR-136 also significantly reduced the apoptosis rate in the hippocampus tissue and inhibited the levels of inflammatory factors. Meanwhile, miR-136 downregulates the expression of Wnt/*β*-catenin signaling pathway-related proteins. However, Wnt pathway activator LiCl could destroy the protective effect of miR-136.

**Conclusion:**

miR-136 could exert its neuroprotective influence on temporal lobe epilepsy rats by inhibiting the Wnt/*β*-catenin signaling pathway.

## 1. Introduction

Epilepsy (Ep) is a chronic brain disorder characterized by recurrent episodes caused by the excessive discharge of a certain part of the neuron group in the brain [1]. The seizures originate in or involve the medial temporal lobe structures, such as the hippocampus. Seizures result from the excessive discharge of abnormal neurons in the brain and can produce severe symptoms, ranging from brief sensory experiences to severe seizures [2]. Among them, temporal lobe epilepsy (TLE) is a subtype of epilepsy, accounting for about one-third of all epilepsies, is the most common focal epilepsy [3], but also the most common refractory epilepsy in adults, often accompanied by progressive etiological pathology and high incidence of drug resistance [4], which is characterized by periodic, unpredictable seizures [5]. Although the understanding of the neuropathology of TLE has made great progress in the past few decades, the complex and nonspecific clinical manifestations of TLE make it easy to be misdiagnosed [6]. In addition, most of the current clinical antiepileptic drugs can only control the symptoms of epileptic seizures, and there is no substantial improvement in the management of TLE [7]. Therefore, exploring the molecular mechanism of the TLE process and finding new antiepileptic drugs have become an important clinical challenge for the treatment of epilepsy [8].

At present, the mechanism of TLE is still not fully understood, but many studies have shown that epileptogenesis involves cascade changes in molecular and cellular networks [9]. At present, studies have shown that microRNA (miRNA) plays a key role in the pathogenesis of some diseases and many biological processes [10]. miRNA is a small noncoding RNA with a length of 18-25 nt produced from genome transcribed RNA with a hairpin structure [11]. Studies have shown that miRNAs play an important role in inflammation and neurological diseases [12]. At present, many studies have pointed out that the imbalance of miRNAs is related to a variety of pathological mechanisms of TLE, and 16 kinds of miRNAs have been found to be inseparably related to epileptic seizures [13]. For example, miR-129-5p inhibits the occurrence of autoimmune encephalomyelitis-associated epilepsy by suppressing HMGB1 expression and inhibiting the TLR4/NF-*κ*B signaling pathway [14]. miR-15a inhibits apoptosis and inflammation in TLE models by downregulating GFAP [15]. miR-136 is a novel miRNA that is significantly underexpressed in a variety of cancers [16–18]. And some scholars have found that miR-136 is enriched in the plasma of Parkinson's patients [19]. In addition, the absence of miR-136 significantly triggers neuropathic pain through neuroinflammatory activation [20]. It shows that miR-136 plays an important role in neurological diseases. However, there are relatively few studies on the effect of miR-136 on TLE, and the specific mechanism of action has not been reported yet. Therefore, this study was conducted to determine the expression of miR-136 in TLE by constructing a rat model of epilepsy induced with pilocarpine. And the effect of miR-136 expression on the hippocampus tissue of rats was detected. Its role and mechanism were explored, aiming to provide new ideas and data basis for the clinical treatment of TLE.

## 2. Materials and Methods

### 2.1. Experimental Animals

Thirty adult male SD rats (190-240 g) were reared at a temperature of 22°C, relative humidity of 60%, and 12 h/12 h in a dark/light environment with free eating and drinking access. Follow-up experiments were carried out after one week of adaptive feeding. The Changzhou Hospital District, 904 Hospital of PLA joint logistics support force (20201027c1200350) Ethics Committee approved this study.

### 2.2. Construction of Rat Temporal Lobe Epilepsy Model

One day in advance, rats were intraperitoneally injected with 127 mg/kg of lithium chloride. Rats were intraperitoneally injected with 1 mg/kg of atropine 1 hour before the injection of pilocarpine. After 30 minutes, rats were intraperitoneally injected with 30 mg/kg of pilocarpine [21]. The severity of seizures was assessed according to the Racine scale. If the rat did not have seizures of grade 4 and above within 30 minutes of the first injection of pilocarpine, the rats were reinjected with the above dose. No seizures after 3 consecutive injections indicated that the model establishment failed. When the seizures lasted for 60 minutes, the rats were given 0.5% diazepam (10 mg/kg) to stop the seizures. The rats were randomly divided into 5 groups (*n* = 6 per group): control group, injected with the same amount of normal saline; Ep group, injected with the same amount of normal saline after successful modeling; NC group, treated with Ep stimulation for 4-6 h, stereotactic injection of agomir NC into the lateral ventricle of Ep rats was done; miR-136 group, after 4-6 h of Ep stimulation, stereotactic injection of miR-136 agomir into the lateral ventricle of Ep rats was done; and miR-136+LiCl group, after 4-6 h of Ep stimulation, Ep rats were stereotactically injected with miR-136 agomir and LiCl into the lateral ventricle. During the intervention treatment, the number and duration of epileptic seizures in each group of rats were recorded. After 7 days, the rats were sacrificed, and their brain tissues were collected.

### 2.3. qRT-PCR

TRizol reagent (Thermo Fisher, USA) was used to extract total RNA from rat hippocampus tissue, and then, NanoDrop was used to detect the concentration and purity of RNA. cDNA was prepared according to the instructions of the reverse transcription kit (Takala, Japan). The cDNA was used to detect the expression level of miR-136 in accordance with the instructions of the SYBR GREEN kit (TaKaRa, Japan), U6 was used as an internal reference control, and the experiment was set with 6 replicates. The experimental data obtained by qRT-PCR was calculated using the 2^-*ΔΔ*Ct^ method to calculate the relative expression of the target gene. The primer sequences used were as follows: miR-136, 5′-ACTCCATTTGTTTTGATGATG-3′ (forward) and 5′-GAACATGTCTGCGTATCTC-3′ (reverse) and U6, 5′-ACCCGTTGAACCCCATTCGTGA-3′ (forward) and 5′-GCCTCACTAAACCATCCAATCGG-3′ (reverse).

### 2.4. H&E Staining

After 48 h of fixation of rat whole brain tissue with 4% paraformaldehyde, the corresponding whole brain regions of the temporal lobe were selected, dehydrated by gradient alcohol, permeabilized with xylene, and embedded in paraffin. The wax block was sectioned with a thickness of 3-4 *μ*m. The sections were then deparaffinized and stained with hematoxylin at room temperature for 5 min, then differentiated with hydrochloric acid alcohol, returned to blue with 1% ammonia by volume fraction, and then washed with tap water and stained with eosin for 30 s. Finally, it was dehydrated with alcohol, treated with xylene, and mounted, and the pathological changes of hippocampal tissue were observed under a biological microscope.

### 2.5. Nissl Staining

After fixing the whole brain tissue of each group of rats with 4% paraformaldehyde for 48 h, they were routinely deparaffinized to water. Rinse 3 times with distilled water, and stain with 1% toluidine for 40 minutes in a 60°C incubator. After washing the dye with distilled water, it was dehydrated, cleared, and then mounted for microscopic inspection. Neuronal damage in the hippocampus was observed, and Nissl body positive cells were quantitatively analyzed.

### 2.6. Enzyme-Linked Immunosorbent Assay (ELISA)

50 mg of rat tissue was taken and placed in a 2 mL homogenization tube; homogenization beads were added along with 1 mL of precooled PBS buffer, homogenized at a 50 Hz frequency for 3 min, and centrifuged at 12000 r/min for 20 min at 4°C to remove cells or cell debris. The supernatant was taken into a new sterile centrifuge tube, and IL-1*β*, IL-6, and TNF-*α* levels in each group of tissues were detected following the instructions of the corresponding ELISA kit (Lianke, China).

### 2.7. Cells Apoptosis

Respectively, take 5 mm^3^ volume of rat hippocampal tissue block, remove the surface fat and fiber, and grind it into a cell suspension in a sterile steel mesh (100 mesh). The cell suspension was filtered through a 200-mesh nylon sieve, and the cell clusters and uncrushed cell clumps were removed and then centrifuged and resuspended to prepare a single-cell suspension. 10 *μ*L of Annexin V-FITC was added along with 10 *μ*L of 20 mg/L PI solution and then incubated at room temperature for 10 min in the dark before adding 500 *μ*L of PBS. Cell apoptosis was detected by flow cytometry.

### 2.8. Western Blot

The hippocampal tissue of each group of rats was used to extract protein with RIPA buffer (Gibco, USA). After measuring the protein concentration with the BCA kit (Thermo Fisher, USA), 20 *μ*g of protein was taken and denatured by boiling in 1× loading buffer. The protein was separated by SDS-PAGE and transferred to the PVDF membrane. After blocking with 5% skimmed milk for 1 h, the membranes were incubated with the primary antibody overnight at 4°C. The membrane was then washed 3 times before the addition of the secondary antibody and incubated at room temperature for 1 h. After washing the membrane three more times, a chemiluminescence reagent was added to develop the protein and placed in the gel imaging system to collect the image. The gray level of the protein bands was analyzed using the ImageJ software. GAPDH was used as the internal reference to calculate the relative protein expression.

### 2.9. Statistical Analysis

The SPSS 25.0 software (SPSS Inc., Chicago, USA) was used for statistical analysis. One-way ANOVA was used to compare multiple groups, and independent sample *t*-test analysis was used to compare two groups. The results were expressed as mean ± standard deviation (SD), and *p* < 0.05 was used as the criterion for judging the significance of the difference.

## 3. Results

### 3.1. miR-136 Ameliorates Epileptic Seizures and Hippocampal Tissue Damage in Epileptic Rats

In order to verify the role of miR-136 in the hippocampus of epileptic rats, the expression of miR-136 in the hippocampus tissue of epileptic rats was first detected. The results showed that the expression of miR-136 was significantly reduced in TLE rats. After overexpression of miR-136, the expression of miR-136 was significantly increased compared with the Ep group, indicating that the overexpression of miR-136 was successful (Figure 1(a)). The effect of miR-136 on the seizures of TLE rats was further monitored. The results showed that after overexpression of miR-136, the number of seizures in rats was significantly reduced, and the duration of each seizure was reduced considerably. While after the addition of the Wnt pathway activator LiCl, the number of seizures in rats was significantly increased compared with the miR-136 group, and the duration was significantly longer (Figures 1(b) and 1(c)).

Further H&E staining results also showed that the nerve cells in the hippocampus of the control group were arranged neatly, with clear edges, round or oval nuclei, clear nucleoli, and lightly stained cytoplasm. The rat hippocampal tissues of the Ep and NC groups had severe neuron damage phenomenon. The cell arrangement was irregular and sparse; the cell gap was enlarged, the number of neurons was obviously reduced, most of the neurons were obviously swollen, the cell body was irregular, the cell protrusion was reduced, and the nucleus was pyknotic, fragmented, and dissolved. After overexpression of miR-136, the number of neurons in the hippocampus tissue was significantly increased compared with that in the NC group. They were arranged more neatly, and histopathological changes were improved. On this basis, after adding LiCl, neurons were damaged, hippocampal neuronal cells were significantly reduced, and the nuclear pyknosis, fragmentation, and dissolution were observed, which was worse than the pathological changes in the miR-136 group (Figure 1(d)). The results of Nissl staining also showed that the neurons in the hippocampus tissue of the control group were arranged neatly, with complete structures, and abundant Nissl bodies were seen. The structure of neurons in the hippocampus tissue of the rats in the Ep and NC groups was disordered, and the number of neuronal cells was significantly reduced, and a large number of Nissl bodies disappeared. The degree of neuron damage in the hippocampus tissue of rats of the miR-136 group decreased, and the number of neurons and Nissl bodies increased significantly compared with the NC group; while the degree of neuron damage in the hippocampus of rats in the miR-136+LiCl group increased, the number of neurons and Nissl bodies was significantly reduced compared with the miR-136 group (Figure 1(e)).

### 3.2. miR-136 Reduces the Inflammatory Response in the Hippocampus of Epileptic Rats and Inhibits Neuronal Cell Apoptosis

The effect of miR-136 on inflammatory response and neurons in TLE rats was further explored by detecting the release of inflammatory factors and cell apoptosis. The results showed that the levels of IL-1*β*, IL-6, and TNF-*α* in the hippocampus tissue of the Ep group were significantly higher than those in the control group, while the levels of IL-1*β*, IL-6, and TNF-*α* in the hippocampus tissue after overexpression of miR-136 was significantly reduced. After adding LiCl, the levels of IL-1*β*, IL-6, and TNF-*α* were significantly higher than those in the miR-136 group (Figure 2(a)). The results of apoptosis detection in the hippocampus tissue also showed that the apoptosis rate and the apoptosis-related protein c-Caspase-3 in the hippocampus tissue of the Ep group were significantly higher than those in the control group, and the expression of Bcl-2 protein was reduced. After overexpression of miR-136, the apoptosis rate and c-Caspase-3 expression in the hippocampus tissue were significantly reduced, and the Bcl-2 protein expression increased. The apoptosis rate and c-Caspase-3 expression in the hippocampus tissue of rats in the miR-136+LiCl group were significantly higher than those of the miR-136 group, and the expression of Bcl-2 protein was significantly reduced (Figures 2(b) and 2(c)).

### 3.3. miR-136 Can Inhibit the Wnt/*β*-Catenin Signaling Pathway in the Hippocampus Tissue of Epileptic Rats

Further studying the mechanism of miR-136 affecting TLE, the results showed that the levels of Wnt/*β*-catenin signaling pathway-related proteins *β*-catenin, Cyclin D1, and c-myc in the hippocampus tissue of the Ep group were significantly higher than those in the control group, while the *β*-catenin, Cyclin D1, and c-myc in the hippocampus tissue were significantly reduced after overexpression of miR-136. Adding LiCl was able to reverse the inhibitory effect of miR-136 on the Wnt/*β*-catenin signaling pathway (Figure 3). This indicates that miR-136 has an inhibitory effect on the Wnt/*β*-catenin signaling pathway in temporal lobe epilepsy.

## 4. Discussion

TLE is the most common type of focal epilepsy, with seizures beginning in the temporal lobe structure [22]. Approximately 30% of TLE patients are ineffective in treatment with antiepileptic drugs to suppress seizures [23, 24]. Therefore, it is necessary to find new therapeutic targets. There are also increasing studies linking miRNAs to TLE. Studies have shown that miR-15a-5p and miR-194-5p in the serum of patients with epilepsy are downregulated, which indicates that miRNAs may be an effective diagnostic marker for epilepsy [25]. Overexpression of miR-136 can also inhibit the development of neuropathic pain [26]. In addition, in spinal cord ischemic injury, miR-136 regulates nerve cell apoptosis by regulating TIMP3 [27]. This shows that miR-136 plays a good role in neuro-related diseases. However, its effect on TLE is unclear. In this study, we found that the expression of miR-136 was downregulated in TLE rats, confirming the involvement of miR-136 in seizures. And overexpression of miR-136 improved the frequency and duration of seizures and ameliorate hippocampal tissue damage in epileptic rats.

Neuronal injury is the main characteristic of neuropathological change in humans and most rodent epilepsy models [28]. At the same time, more and more studies have shown the relevance of neuroinflammation in the pathophysiology of epilepsy, which contributes to neuronal damage [29]. Clinical studies have also shown that the levels of proinflammatory cytokines (such as IL-6, TNF-*α*, and IL-1*β*) in the serum or cerebrospinal fluid of patients with epilepsy are elevated [30]. This study also showed that miR-136 could reduce the inflammatory response and neuronal apoptosis in the hippocampus tissue of epileptic rats. This suggests that upregulation of miR-136 expression may be a potential way to treat TLE.

The Wnt/*β*-catenin signaling pathway can affect various cellular processes, such as proliferation, differentiation, apoptosis, and cell motility [31]. When the Wnt/*β*-catenin signaling pathway is abnormal, it can lead to the occurrence and development of diseases and affect the occurrence and progression of human cancer or other diseases [32]. Studies have shown that miR-136 can target PMEL through the Wnt signaling pathway to inhibit the proliferation, apoptosis, and epithelial-mesenchymal transition biological processes of melanoma cells [33]. miR-136 can also inhibit the proliferation and invasion of colon cancer cells by targeting LRH-1/Wnt signaling pathway [34]. This suggests that miR-136 mediates disease onset and progression through regulating the Wnt/*β*-catenin signaling pathway. In the present study, it was also found that miR-136 overexpression inhibited the expression of *β*-catenin, Cyclin D1, and c-myc in the hippocampus tissue of epileptic rats. It is suggested that miR-136 exerts its biological functions in the TLE by inhibiting the Wnt/*β*-catenin signaling pathway activity. However, the specific mechanism of whether miR-136 acts through the regulation of target genes mediating the Wnt/*β*-catenin signaling pathway in the TLE needs to be further explored.

## 5. Conclusion

In summary, miR-136 was downregulated in the hippocampus of epileptic rats. Overexpression of miR-136 could inhibit Wnt/*β*-catenin signaling pathway activation, inhibit neuronal death, and reduce inflammation, thereby reducing the seizure frequency and duration of epileptic rats and affecting the occurrence of TLE. This result suggested that miR-136 might be a new biomarker and therapeutic target for TLE.

## Figures and Tables

**Figure 1:** The effect of miR-136 on seizures and hippocampus tissue in temporal lobe epilepsy rats. (a) qRT-PCR was used to detect the expression of miR-136 in the hippocampus of each group of rats. (b) The frequency of seizures in each group of rats. (c) The duration of seizures in each group of rats. (d) H&E staining was used to observe the pathological changes of the hippocampus tissue of rats of each treatment group. (e) Nissl staining was used to observe the neuron death of the hippocampus tissue of the rats in each treatment group. *N* = 6 per group. ^∗∗^*p* < 0.01 vs. control group, ^##^*p* < 0.01 vs. NC group, and ^&&^*p* < 0.01 vs. miR-136 group. EP: epilepsy; NC: agomir NC; miR-136: miR-136 agomir; miR-136+LiCl: miR-136 agomir and Wnt pathway activator.

**Figure 2:** The effect of miR-136 on hippocampal tissue inflammatory response and neuronal apoptosis in temporal lobe epilepsy rats. (a) ELISA was used to detect the levels of IL-1*β*, IL-6, and TNF-*α* in the hippocampus tissue of each group of rats. (b) Flow cytometry was used to detect the apoptosis of neurons in the hippocampus tissue of each treatment group. (c) Western blot was used to detect the expression of apoptosis-related proteins c-Caspase-3 and Bcl-2. *N* = 6 per group. ^∗∗^*p* < 0.01 vs. control group, ^##^*p* < 0.01 vs. NC group, and ^&&^*p* < 0.01 vs. miR-136 group.

**Figure 3:** The effect of miR-136 on the Wnt/*β*-catenin signaling pathway in the hippocampus tissue of epileptic rats. *N* = 6 per group. ^∗^*p* < 0.05 and ^∗∗^*p* < 0.01 vs. control group, ^#^*p* < 0.05 and ^##^*p* < 0.01 vs. NC group, and ^&^*p* < 0.05 and ^&&^*p* < 0.01 vs. miR-136 group.

## Data Availability

The data used to support the findings of this study are available from the corresponding author upon request.
